RETRACTED

# Overexpression of TGFβ1 in murine mesenchymal stem cells improves lung inflammation by impacting the Th17/Treg balance in LPS-induced ARDS mice

**DOI:** 10.1186/s13287-020-01826-0

**Published:** 2020-07-22

**Authors:** Jianxiao Chen, Xiwen Zhang, Jianfeng Xie, Ming Xue, Ling Liu, Yi Yang, Haibo Qiu

**Affiliations:** Jiangsu Provincial Key Laboratory of Critical Care Medicine, Department of Critical Care Medicine, School of Medicine, Zhongda Hospital, Southeast University, 87 Dingjiaqiao Road, Nanjing, 210009 People’s Republic of China

**Keywords:** Acute respiratory distress syndrome, Mesenchymal stem cells, TGFβ1, Th17/Treg

## Abstract

**Background:**

T helper 17 cells (Th17)/regulatory T cells (Treg), as subtypes of CD4^+^ T cells, play an important role in the inflammatory response of acute respiratory distress syndrome (ARDS). However, there is still a lack of effective methods to regulate the differentiation balance of Th17/Treg. It was proven that mesenchymal stem cells (MSCs) could regulate the differentiation of CD4^+^ T cells, but the mechanism is still unclear. TGFβ1, a paracrine cytokine of MSCs, could also regulate the differentiation of Th17/Treg but is lowly expressed in MSCs. Therefore, mouse MSCs (mMSCs) overexpressing TGFβ1 were constructed by lentivirus transduction and intratracheally transplanted into LPS-induced ARDS mice in our study. The aim of this study was to evaluate the therapeutic effects of mMSCs overexpressing TGFβ1 on inflammation and immunoregulation by impacting the Th17/Treg balance in LPS-induced ARDS mice.

**Methods:**

mMSCs overexpressing TGFβ1 were constructed using lentiviral vectors. Then, mouse bone-marrow-derived MSCs (mBM-MSC) and mBM-MSC-TGFβ1 (mBM-MSC overexpressing TGFβ1) were transplanted intratracheally into ARDS mice induced by lipopolysaccharide. At 3 and 7 days after transplantation, the mice were sacrificed, and the homing of the mMSCs was assayed by ex vivo optical imaging. The relative numbers of Th17 and Treg in the lungs and spleens of mice were detected by FCM. IL-17A and IL-10 levels in the lungs of mice were analysed by western blot. Permeability and inflammatory cytokines were evaluated by analysing the protein concentration of BALF using ELISA. Histopathology of the lungs was assessed by haematoxylin and eosin staining and lung injury scoring. Alveolar lung fibrosis was assessed by Masson’s trichrome staining and Ashcroft scoring. The mortality of ARDS mice was followed until 7 days after transplantation.

**Results:**

The transduction efficiencies mediated by the lentiviral vectors ranged from 82.3 to 88.6%. Overexpressing TGFβ1 inhibited the proliferation of mMSCs during days 5–7 (*p* < 0.05) but had no effect on mMSC differentiation or migration (*p* > 0.05). Compared to that in the LPS + mBM-MSC-NC group mice, engraftment of mMSCs overexpressing TGFβ1 led to much more differentiation of T cells into Th17 or Treg (*p* < 0.05), improved permeability of injured lungs (*p* < 0.05) and ameliorative histopathology of lung tissue in ARDS mice (*p* < 0.05). Moreover, IL-17A content was also decreased while IL-10 content was increased in the LPS + mBM-MSC-TGFβ1 group compared with those in the LPS + mBM-MSC-NC group (*p* < 0.05). Finally, mMSCs overexpressing TGFβ1 did not aggravate lung fibrosis in ARDS mice (*p* > 0.05).

RETRACTED

**Conclusion:**

MSCs overexpressing TGFβ1 could regulate lung inflammation and attenuate lung injuries by modulating the imbalance of Th17/Treg in the lungs of ARDS mice.

## Background

Acute respiratory distress syndrome (ARDS), which was initially defined 52 years ago as a multifactorial syndrome of severe lung injury [1], is characterised by hypoxaemia, loss of lung compliance, and pulmonary oedema, which can in some instances progress to multiple organ failure [2]. ARDS can develop in response to multiple predisposing factors, including pneumonia, systemic infection, and major surgery or multiple traumas [3], and results in death in 30–45% of cases [4].

In the past 50 years, considerable progress has been made in understanding the pathology of ARDS, and the development of ARDS is strongly associated with a disordered immune response in the lung [5]. In previous studies, CD4^+^ T cells, as an important component of adaptive immune cells, were significantly activated in the early stage of ARDS, and the differentiation of T helper 17 cells (Th17)/regulatory T cells (Treg) played an important role in the development of ARDS [5]. Th17 can release many inflammatory cytokines that mediate the acute inflammatory response [6]. Treg, as important immunosuppressive cells, can also be activated in ARDS, and the transplantation of Treg into an ARDS model mice may reduce the levels of proinflammatory cytokines in the alveoli [7] and inhibit neutrophil apoptosis and fibrocyte recruitment [8]. In addition, the differentiation balance of Th17/Treg is an independent predictor for 28-day mortality in patients with ARDS [9]. Thus, there is still a lack of effective methods to regulate the differentiation balance of Th17/Treg.

Our previous study proved that mesenchymal stem cells (MSCs), with their multipotency and immunoregulation properties, could significantly improve inflammation and repair lung injuries in ARDS mice [10]. The mechanism of their immunological regulation may be related to the modulation of T cell expansion [11]. It has also been confirmed in a recently published study that MSCs could regulate the imbalance of Th17/Treg, which is regulated by antigen-stimulated costimulatory molecules, antigen-presenting cells, cytokines, and intracellular signals [11]. TGFβ1, an important cytokine that regulates the differentiation of Th17/Treg [12], is expressed at low levels in MSCs, which was proven by our preliminary data. Thus, overexpression of TGFβ1 is expected to further optimise MSC treatment for immunoregulation.

RETRACTED

Therefore, the aim of this study was to evaluate the effect of mouse MSCs (mMSCs) overexpressing TGFβ1 on inflammation and immunoregulation in LPS-induced ARDS mice.

## Materials and methods

### Cell culture

mMSCs isolated from the bone marrow of C57BL/6 mice (mBM-MSC) were purchased from Cyagen Biosciences, Inc. (Guangzhou, China), and 293 T cells were supplied by Zoonbio Biotechnology Co., Ltd. (Nanjing, China). The mBM-MSC were identified by detecting cell surface phenotypes and their multipotent potential for differentiation along the adipogenic, osteogenic, and chondrogenic lineages as previously described [13, 14].

Either mBM-MSC or 293 T cells were cultured in a 1:1 mix of Dulbecco’s modified Eagle’s medium/nutrient mixture F-12 (DMEM/F12) (Wisent, Inc., St-Bruno, Montreal, Quebec, Canada) containing 10% FBS (Wisent, Inc.) and 1% antibiotic-antimycotic (streptomycin, penicillin and amphotericin B; Wisent, Inc.), incubated at 37 °C in a humidified atmosphere of 5% CO_2_ and passaged every 3–4 days by 0.25% trypsin-ethylenediaminetetraacetic acid (EDTA; Gibco, Carlsbad, CA, USA) when they reached approximately 80% confluence. Passages between 5 and 10 were used for the experimental protocols.

### Recombinant lentivirus vector construction and packaging

The full-length coding sequence (CDS) of mouse TGFβ1 was transferred into the CMV promoter-dependent lentivirus vector PDS159_pL6.3-CMV-GFPa1-IRES-MCS (Zoonbio Biotechnology Co., Ltd.). Subsequently, the lentivector CL721-pL6.3-CMV-GFPa1-IRES-mus-TGF-β (overexpressing TGFβ1), which co-expresses enhanced green fluorescent protein (eGFP) and TGFβ1, was obtained, and the empty vector CL721-pL6.3-CMV-GFPa1-IRES was used as an empty vector control. Then, the recombinant plasmids CL721-pL6.3-CMV-GFPa1-IRES-mus-TGF-β and CL721-pL6.3-CMV-GFPa1-IRES were separately co-transfected with packaging plasmids into 293 T cells at the indicated concentrations using Lipofectamine 2000 (Invitrogen Life Technologies) according to the manufacturer’s instructions, producing the lentivirus LV402-pL6.3-CMV-GFPa1-IRES-mus-TGF-β and the negative control PDS019.

### Lentiviral vector transduction and eGFP reporter gene detection

The mBM-MSC (1 × 10^6^/well seeded in six-well cell culture plates) were transduced with viral supernatant at a multiplicity of infection (MOI) of 160:1 for 24 h. Then, the stable cell lines were harvested after selection using blasticidin (BSD; InvivoGen) at the minimal lethal concentration (6 μg/mL) as previously described [15] and cultured in normal culture medium for 20 passages after transduction. Finally, the transduction efficiency of mBM-MSC and the percentage of eGFP-positive cells were evaluated by fluorescence microscopy and flow cytometry (FCM) analysis using a FACSCalibur flow cytometer (Becton-Dickinson, Franklin Lakes, NJ, USA).

RETRACTED

### Cell surface phenotype detection

The cells were also identified by detecting cell surface phenotypes after lentivirus transduction. Fluorescein conjugated monoclonal antibodies, including CD29, CD34, CD44, CD105, and CD45, and the respective isotype controls were purchased from Becton-Dickinson (Franklin Lakes, NJ, USA). FCM analysis was performed with fluorescence-activated cell sorting analysis.

### RNA isolation and quantitative real-time PCR (qRT-PCR)

Total RNA was isolated from the cells and tissues using TRIzol reagent (Invitrogen, Austin, TX, USA) according to the manufacturer’s protocol, and the purity of the RNA (260/280 nm absorbance ratio of 1.8–2.2) was assessed by a spectrophotometer (Tecan, Switzerland). Reverse transcription was completed using a RevertAid First Strand cDNA Synthesis Kit (Thermo Scientific) with 1 mg of RNA according to the manufacturer’s instructions. qRT-PCR was performed using a CFX96™ Real-Time system (Bio-Rad). Relative changes in gene expression were normalised to the expression of actin and calculated by the 2(−ΔΔCt) method. The primer sequences used for PCR amplification in our study were designed based on the sequences of the genomic clones and are as follows:

**Table:** 

Gene	Primer	Primer sequence	PCR amplified product (bp)
Actin	Forward	5′-AGAGGGAAATCGTGCGTGAC-3′	195
	Reverse	5′-CCATACCCAAGAAGGAAGGCT-3′	
GADPH	Forward	5′-TGTGTCCGTCGTGGATCTGA-3′	150
	Reverse	5′-TTGCTGTTGAAGTCGCAGGAG-3′	
TGFβ1	Forward	5′-GACTCTCCACCTGCAAGACC-3′	100
	Reverse	5′-GGACTGGCGAGCCTTAGTTT-3′	
Collagen I	Forward	5′-GTGTTTCCTGTGCTACTG-3′	132
	Reverse	5′-TCTTTCTCCTCTCTGACC-3′	
α-SMA	Forward	5′-CCTCGCCTCTACCCCTTA-3′	120
	Reverse	5′-ATTCGCTTGCCTTTGCTT-3′	

### Western blot analysis

To evaluate the TGFβ1 concentration in mBM-MSC, the total cellular protein was extracted by RIPA lysis buffer (Beyotime Institute of Biotechnology, Haimen, China) containing an antiprotease cocktail (1 mmol/L PMSF, 1 mmol/L NaF and 1 mmol/L Na_3_VO_4_; US Biological Inc., Swampscott, MA, USA) according to the manufacturer’s instructions, quantified by a BCA protein assay kit (Beyotime), separated by sodium dodecyl sulfate-polyacrylamide gel electrophoresis (SDS-PAGE) (10%), electro-transferred to PVDF membranes (Millipore, Bedford, MA, USA), and then incubated with primary antibodies against TGFβ1 (1:5000 dilution; Abcam Incorporated, Cambridge, MA) or β-actin (1:3000 dilution; Abcam Incorporated, Cambridge, MA) at 4 °C overnight. The blots were washed three times with TBST and then incubated for 1 h at room temperature with goat anti-rabbit IgG conjugated with horseradish peroxidase (1:5000 dilution; Zoonbio Biotechnology). Immunoreactive complexes were visualised by chemiluminescence reagents (Thermo Fisher Scientific Inc., Waltham, MA, USA), and immunoreactive bands were obtained using a chemiluminescence imaging system (BioshineChemiQ4800 mini; Ouxiang, Shanghai, China). Finally, the intensity of those bands was analysed by Image J software (NIH, USA).

RETRACTED

### Protein concentration in culture medium

mBM-MSC, mBM-MSC-NC, and mBM-MSC-TGFβ1 were seeded in a 12-well plate at a density of 1 × 10^5^ cells per well. After 12 h, the culture medium was changed, and mBM-MSC were cultured in an incubator at 37 °C and 5% CO_2_ for 24 h. The culture medium was then collected, and TGFβ1 protein levels in the culture medium were quantified using an enzyme-linked immunosorbent assay (ELISA) kit (Abcam, USA) according to the manufacturer’s instructions.

### Cell proliferation assay

Cell Counting Kit-8 (CCK-8; Beyotime Institute of Biotechnology, Haimen, China) assays were used to further investigate the effects of overexpressing TGFβ1 on mBM-MSC proliferation according to the manufacturer’s instructions. Briefly, cells were seeded in 96-well plates at 2 × 10^3^ cells per well in 100 μL of growth medium. After staining with CCK-8 (10 μL per well), the cells were incubated for 4 h at 37 °C. Absorbance was assessed at 450 nm with a microplate reader (Tecan, Switzerland).

### Multidifferentiation of mMSCs after gene transduction

For osteogenic differentiation, the cells were seeded in 6-well plates and cultured in 2 mL of DMEM/F12 supplemented with 10% FBS. When the cells reached approximately 80–90% confluence, they were switched to C57BL/6 mMSC osteogenic differentiation medium (Cyagen Biosciences, Inc., Guangzhou, China) for 2–3 weeks. Calcium deposition was assessed by staining the cells with 40 mM Alizarin Red S solution at room temperature for 10 min.

For adipocytic differentiation, when reaching confluence, the cells were treated with mMSCs adipogenic differentiation basal medium A (Cyagen Biosciences, Inc., Guangzhou, China) for 3 days, followed by exchange with mMSCs adipogenic differentiation basal medium B (Cyagen Biosciences, Inc., Guangzhou, China) for 24 h and then switching back to basal medium A. After five to six cycles, the cells were cultured in basal medium B for 3 days until their lipid vacuoles enlarged. To assess the accumulation of neutral lipid vacuoles, the cells were stained with filtered Oil Red O solution for 10 min at room temperature, and the incorporated Oil Red O was extracted by adding 1 mL of isopropanol to each well at room temperature for 15 min.

RETRACTED

For chondrogenic differentiation, 2.5 × 10^5^ cells were centrifuged in a 15 mL tube at 150×*g* for 5 min to form a pellet. Chondrogenic differentiation was achieved by the three-dimensional culture method and C57BL/6 mMSCs chondrogenic differentiation medium (Cyagen Biosciences, Inc., Guangzhou, China). After 28 days, the pellets were embedded in paraffin and then fixed in dimethylbenzene and ethanol. Five-micrometre sections were cut and stained with Alcian blue to determine the polysaccharide accumulation.

### In vitro scratch assay

The horizontal migration of cells was determined by the in vitro scratch assay. Cells were seeded in six-well culture plates. After reaching approximately 100% confluence, a scratch was made with a 10-μL sterile pipette tip. Then, the cells were cultured in serum-free DMEM/F12 for another 12 h. The images of the wound area were recorded by a light microscope immediately after scratching and 12 h later. The horizontal migration ability of the cells was quantified by measuring the wound area in each group by Image J analysis software [13].

### Transwell migration assay

The vertical migration of cells was determined by the Transwell migration assay. Transwell inserts (6.5 mm diameter and 8 mm pore size; Millipore) that were seeded with 2 × 10^4^ cells in 100 μL of serum-free DMEM/F12 were loaded into lower chambers with 600 μL of DMEM/F12 supplemented with 10% FBS. After incubation for 12 h, the cells remaining on the upper surface of the inserts were removed with cotton swabs, and the cells that had migrated to the lower surface were stained with crystal violet (Beyotime Institute of Biotechnology, Haimen, China) for 20 min. The stained cells from four randomly chosen areas were measured under a light microscope [13].

### Ethics statement

All animal experiments in this study were performed in accordance with the Guide for the Care and Use of Laboratory Animals and were approved by the Institutional Animal Care and Use Committee of Southeast University. Wild-type (WT) C57BL/6 mice aged 6–8 weeks were purchased from the Laboratory Animal Centre (Shanghai, China). Mice were housed in individual microisolator cages under specific pathogen-free conditions with free access to water and chow.

RETRACTED

### Murine model of lipopolysaccharide-induced acute respiratory distress syndrome

After anaesthetization with an intraperitoneal injection of pentobarbital at 50 mg/kg, mice were subjected to intratracheal (i.t.) administration of LPS (2 mg/kg, *Escherichia coli* serotype 0111:B4; Sigma-Aldrich, St Louis, MO, USA) dissolved in 20 μL of sterile normal saline (NS). Sham operation was performed in a similar manner with the same volume of only 0.9% NS instead of LPS. Then, the mice recovered until fully awake in a 100% oxygen chamber.

### Experimental protocol

The mice were randomly divided into five groups as follows: the control group, mice that received phosphate-buffered saline (PBS) intratracheally 4 h after i.t. administration of 0.9% NS; the ARDS group, mice that received PBS intratracheally 4 h after LPS challenge; the LPS + mBM-MSC group, mice that received WT mBM-MSC (2 × 10^5^ cells per mouse) intratracheally; the LPS + mBM-MSC-NC group, mice that received mBM-MSC-NC (normal control, 2 × 10^5^ cells per mouse) intratracheally; and the LPS + mBM-MSC-TGFβ1 group, mice that received mBM-MSC-TGFβ1 (overexpressing TGFβ1, 2 × 10^5^ cells per mouse) intratracheally. The mice were sacrificed at 1, 3, or 7 days after mBM-MSC injection, and the lung lobes were collected for further analysis.

### Preparation of lung tissue lymphocytes and flow cytometry analysis

After the mice were sacrificed, 5 mL of PBS/0.6 mM EDTA was injected into the right ventricular cannula for lung perfusion. The lung was then isolated from the surrounding tissue and added to medium containing digestive enzymes (RPMI 1640, 20 mM HEPES, 10% FCS, 175 U/mL collagenase, 75 U/mL DNAse I, 0.2 U/mL pancreatic elastase, 35 U/mL hyaluronidase, 100 IU/mL penicillin, and 100 mg/mL streptomycin) for incubation for 45 min at 37 °C. The resulting suspension was passed three times through a 19-gauge needle to break up clumps and then through a 40-mm filter to remove debris. The leukocytes were enriched by discontinuous Percoll gradient centrifugation and recovered at the interface between 40% Percoll and 70% Percoll layers [16].

The following antibodies (Miltenyi, USA) were used for surface and nuclear staining: FITC-labelled anti-CD4, APC-labelled anti-CD25, PE-labelled anti-Foxp3, and PE-labelled anti-RORγt. For the analysis of Treg, cells were incubated with the surface marker antibodies FITC-anti-CD4 and APC-anti-CD25, followed by fixation and permeabilization with Foxp3-staining buffer (Miltenyi) and intracellular staining with PE-labelled anti-Foxp3. To detect the phenotypes of Th17 cells in the lungs, cells were incubated with the surface markers FITC-anti-CD4 and APC-anti-CD25. Then, the cells were fixed and permeabilized using RORγt-staining buffer (Miltenyi), followed by intracellular staining with PE-labelled anti-RORγt.

RETRACTED

### Protein concentration in the lungs and bronchoalveolar lavage fluid

To analyse the expression of IL-17A, IL-10, and occludin in the lungs after transplantation, total protein lysates were extracted by RIPA lysis buffer (Beyotime) from left lung lobes (*n* = 3 per group at each time-point) and measured by western blot as previously described. The PVDF membranes were incubated with primary antibodies against IL-17A (1:5000 dilution, Abcam), IL-10 (1:5000 dilution, Abcam), occludin (1:5000 dilution; Abcam), or β-actin (1:3000 dilution; Abcam Incorporated, Cambridge, MA).

Bronchoalveolar lavage fluid (BALF) was collected by flushing 1 mL of ice-cold PBS back and forth three times through a tracheal cannula as previously described [14, 15]. After centrifugation at 800×*g* for 10 min, total protein (TP), albumin (ALB), tumour necrosis factor-α (TNF-α), and IL-1β and IL-6 concentrations in the BALF were measured by ELISA kits (Cusabio Biotech, Wuhan, China; Excell Bio, Shanghai, China).

### Labelling and tracing of mesenchymal stem cells

WT mBM-MSC, mBM-MSC-NC, and mBM-MSC-TGFβ1 were labelled with CellVue NIR815 dye (eBioscience Inc., San Diego, CA, USA) according to the manufacturer’s instructions. Then, NIR815-labelled cells (5 × 10^5^ cells) were directly administered into the trachea of the mice in different groups according to the protocol. After 1, 3, and 7 days post-transplantation, three mice at each time point were sacrificed, and ex vivo lungs were imaged using a Maestro in vivo optical imaging system (excitation = 786 nm, emission = 814 nm, and 4000 ms exposure time; Caliper Life Sciences, MA, Boston, USA) [15, 17]. The autofluorescence spectra were then unmixed based on their spectral patterns using Maestro 2.4 software (Caliper Life Sciences). The fluorescence intensity of the lungs was measured by placing the regions of interest (ROIs) on the lungs, and the signals were analysed based on the total fluorescence counts of the ROIs.

### Evaluation of lung oedema

Lung oedema was evaluated using the ratio of lung wet weight to body weight (LWW/BW), which was measured as previously described [17]. Briefly, the whole lung was removed and cleared of all extrapulmonary tissues, and the LWW/BW was calculated based on the values of the lung wet weight and the body weight (mg/g).

### Lung histopathology analysis

The right lung lobes (*n* = 3 for each group at each time-point) were collected and fixed in 4% paraformaldehyde, embedded in paraffin, and sliced into 5 μm sagittal sections. After staining with a haematoxylin and eosin staining kit (Beyotime Institute of Biotechnology, Haimen, China), the slices were then viewed by a pathologist based on ten randomly selected high-power fields (× 400) in each section according to oedema, alveolar and interstitial inflammation, alveolar and interstitial haemorrhage, atelectasis, and necrosis, which was graded on a 0- to 4-point scale (0, no injury; 1, injury in 25% of the field; 2, injury in 50% of the field; 3, injury in 75% of the field; and 4, injury throughout the entire field). The total lung injury score was calculated as the sum of these scores, which has been described previously [14, 15, 17].

RETRACTED

### Lung fibrosis analysis

The lung sections were stained sequentially with Weigert’s iron haematoxylin solution, Biebrich scarlet-acid fuchsin solution, and aniline blue solution, and a blue signal indicated positive staining for collagen. The criteria of Ashcroft were used [15, 17] to assess lung fibrosis, which was quantified based on the findings in ten randomly selected high-power fields (× 400) for each slide by histopathologists blinded to the protocol. Collagen-I and α-SMA mRNA expression in lung tissues was measured by RT-PCR.

### Statistical analysis

The data are presented as the means ± standard deviations (SDs). Statistical analyses were performed using SPSS 26.0 (SPSS Inc., Chicago, IL, USA) and GraphPad Prism 8 (GraphPad Software, La Jolla, California USA). Comparisons among multiple groups were performed by one-way ANOVA followed by Bonferroni’s post hoc test if the data were normally distributed. Kaplan-Meier curves were used to describe the survival rate of mice in each group, and log-rank tests were performed to analyse the significance of differences. A *p* value < 0.05 was considered statistically significant.

## Results

### The efficiency of lentiviral vector-mediated TGFβ1 overexpression in mMSCs

The transduction efficiency, which was reflected by the eGFP-positive cell ratio in our study, mediated by the lentiviral vectors after 20 passages was detected by fluorescence microscopy and FCM analysis. The transduction efficiencies of cells overexpressing TGFβ1 were 82.3–88.6% (Fig. 1a, b). TGFβ1 mRNA levels in mMSCs were detected by qRT-PCR. TGFβ1 mRNA expression was significantly higher in the mBM-MSC-TGFβ1 group than in the mBM-MSC-NC group (*p* < 0.0001). However, there was no significant difference between the mBM-MSC and mBM-MSC-NC groups (*p* > 0.05, Fig. 1c). Secreted TGFβ1 levels in the culture media of mMSCs were significantly higher in the mBM-MSC-TGFβ1 group than in the mBM-MSC-NC group (*p* < 0.0001, Fig. 1d). The western blot analysis also showed similar results for TGFβ1 protein expression in mMSCs (Fig. 1e). Thus, lentivirus-mediated TGFβ1 transduction was stable and efficient.

RETRACTED

**Fig. 1:** Measurement of TGFβ1 expression in mMSCs after lentiviral vector transduction. **a** mBM-MSC, mBM-MSC-NC, and mBM-MSC-TGFβ1 were cultured for 20 passages and observed by light microscopy (top) and fluorescence microscopy with green fluorescent protein (bottom), × 200. **b** The percentage of GFP-positive cells was analysed by flow cytometry at passage 20 after transduction. **c** Evaluation of TGFβ1 mRNA expression in mMSCs after transduction (*n* = 3; *p < 0.0001 vs. mBM-MSC-NC). **d** Evaluation of secreted TGFβ1 in the culture medium of mMSCs after transduction by ELISA (*n* = 3; *p < 0.0001 vs. mBM-MSC-NCs). **e** Detection by western blot analysis of TGFβ1 protein levels in mMSCs after transduction (*n* = 3; *p < 0.0001 vs. mBM-MSC-NCs). mMSCs, mouse mesenchymal stem cells; NC, normal control

In this study, calcium deposition examined by Alizarin Red S staining, lipid accumulation by Oil Red O staining, and polysaccharide accumulation by Alcian blue staining experiment were used to evaluate the multidifferentiation of mMSCs after gene transduction. TGFβ1 transduction did not change the multipotential differentiation ability of mMSCs (Fig. 2b).

**Fig. 2:** The effects of overexpressing TGFβ1 on the proliferation, differentiation, and migration of mMSCs. **a** The effects of overexpressing TGFβ1 on the proliferation of mMSCs. The growth curves of the cells after transduction for 7 days were evaluated by CCK-8 assay (*n* = 3; *p < 0.05 vs. mBM-MSC-NCs). **b** The effects of overexpressing TGFβ1 on the multipotential differentiation of mMSCs. Calcium deposition (top), accumulation of neutral lipid vacuoles (middle), and polysaccharide accumulation (bottom) were detected respectively, × 200. **c** The effects of overexpressing TGFβ1 on the horizontal migration of mMSCs. The wound areas were photographed at 0 and 12 h and quantified by measuring the wound area in each group, × 100 (*n* = 3). **d** The effects of overexpressing TGFβ1 on the vertical migration of mMSCs. The migrated cells on the lower surface of Transwell inserts were stained with crystal violet and measured under a light microscope from four randomly chosen areas, × 100 (*n* = 3). CCK-8, Cell Counting Kit-8; mMSCs, mouse mesenchymal stem cells; NC, normal control

According to FCM analysis, CD29, CD44, and CD105 were positive while CD34 and CD45 were negative on mBM-MSC-TGFβ1, which was in line with the surface markers of mBM-MSC (Supplementary Figure 1).

### Effects of overexpressing TGFβ1 on the proliferation of mMSCs

A CCK-8 assay was used to evaluate the effects of overexpressing TGFβ1 on cell proliferation. By comparing different growth curves, it was found that overexpression of TGFβ1 significantly decreased cell proliferation in the mBM-MSC-TGFβ1 group compared to that in the mBM-MSC-NC group from days 5 to 7 (*p* < 0.05). There was no significant difference between the mBM-MSC and mBM-MSC-NC groups (*p* > 0.05, Fig. 2a).

RETRACTED

### Effects of overexpressing TGFβ1 on the migration of mMSCs

The scratch assay and Transwell assay were used to indicate the horizontal and vertical migration abilities of mMSCs. There were no significant differences in the wound areas in the scratch assay among the mBM-MSC, mBM-MSC-NC, and mBM-MSC-TGFβ1 groups after 12 h of incubation (*p* > 0.05, Fig. 2c). Similar results were also detected in the Transwell assay. No significant differences among the groups were observed (*p* > 0.05, Fig. 2d).

### Effects of overexpressing TGFβ1 on the graft retention of mMSCs in the lung after lipopolysaccharide challenge

To track intrapulmonary mMSCs, ex vivo NIR imaging was performed on the lungs at 1, 3, and 7 days after mMSCs administration. There were no significant differences in the fluorescent counts of ROIs among the groups (*p* > 0.05, Fig. 3a, b).

**Fig. 3:** The effect of overexpressing TGFβ1 on the graft retention of mMSCs in the lungs after LPS challenge. **a** Typical ex vivo NIR images of injured lungs from mice at 1, 3, and 7 days after mMSCs administration. **b** Average signal from ex vivo NIR imaging of injured lungs from mice at 1, 3, and 7 days after mMSCs administration (*n* = 3). mMSCs, mouse mesenchymal stem cells; NIR, near-infrared fluorescence

### Mesenchymal stem cells overexpressing TGFβ1 inhibited lung inflammation in lipopolysaccharide-induced ARDS mice

The differentiation of Th17 and Treg in the lungs of LPS-induced ARDS mice was detected by FCM. At 3 days after mMSCs transplantation, the number of CD4^+^ T cells in the lungs increased significantly in the LPS + mBM-MSC, LPS + mBM-MSC-NC, and LPS + mBM-MSC-TGFβ1 groups compared with that in the ARDS group (*p* < 0.05, Fig. 4a). Meanwhile, the proportion of Th17 significantly decreased in the LPS + mBM-MSC and LPS + mBM-MSC-NC groups compared to that in the ARDS group (*p* < 0.05) but significantly increased in the LPS + mBM-MSC-TGFβ1 group compared to that in the LPS + mBM-MSC-NC group (*p* < 0.05) but was still lower than that in the ARDS group (*p* < 0.05, Fig. 4b). In addition, the proportion of Treg in the LPS + mBM-MSC and LPS + mBM-MSC-NC groups was significantly lower than that in the ARDS group (*p* < 0.05), and the proportion in the LPS + mBM-MSC-TGFβ1 group was significantly higher than that in the LPS + mBM-MSC-NC group (*p* < 0.05) and even higher than that in the ARDS group (*p* < 0.05, Fig. 4c). Moreover, the Th17/Treg ratio in the LPS + mBM-MSC and LPS + mBM-MSC-NC groups was significantly lower than that in the ARDS group (*p* < 0.05), and that in the LPS + mBM-MSC-TGFβ1 group was even lower than that in the LPS + mBM-MSC-NC group (*p* < 0.05, Fig. 4d).

RETRACTED

**Fig. 4:** The effect of mMSCs overexpressing TGFβ1 on the differentiation of CD4^+^ T cells in the lungs of ARDS mice at 3 d after mMSC transplantation. **a**–**d** The differentiation of Th17 and Treg in the lungs of LPS-induced ARDS mice was detected by flow cytometry (*n* = 3, *p < 0.05 compared with the control group; ^#^*p* < 0.05 compared with the ARDS group; ^δ^*p* < 0.05 compared with the LPS + mBM-MSC-NC group). **e** Representative flow cytometry analysis was shown for each treatment group. ARDS, acute respiratory distress syndrome; mMSCs, mouse mesenchymal stem cells; NC, normal control

In addition, similar results were also observed at 7 days after mMSCs transplantation. Compared with that in the lungs of the ARDS group, the number of CD4^+^ T cells increased significantly in the lungs of the LPS + mBM-MSC, LPS + mBM-MSC-NC, and LPS + mBM-MSC-TGFβ1 groups (*p* < 0.05, Fig. 5a). At the same time, the proportion of Th17 in the LPS + mBM-MSC and LPS + mBM-MSC-NC groups decreased significantly compared to that in the ARDS group (*p* < 0.05), and the proportion in the LPS + mBM-MSC-TGFβ1 group decreased further relative to that in the LPS + mBM-MSC-NC group (*p* < 0.05, Fig. 5b). In addition, the proportion of Treg in the LPS + mBM-MSC and LPS + mBM-MSC-NC groups was significantly lower than that in the ARDS group (*p* < 0.05), and the proportion in the LPS + mBM-MSC-TGFβ1 group was slightly higher than that in the LPS + mBM-MSC-NC group (*p* < 0.05) but still lower than that in the ARDS group (*p* < 0.05, Fig. 5c). The Th17/Treg ratio in the LPS + mBM-MSC-TGFβ1 group was significantly lower than that in the LPS + mBM-MSC-NC group (*p* < 0.05, Fig. 5d). It was suggested that mMSCs overexpressing TGFβ1 could further regulate the differentiation of Th17 and Treg and improve the balance of Th17/Treg in the lungs of ARDS mice.

**Fig. 5:** The effect of mMSCs overexpressing TGFβ1 on the differentiation of CD4^+^ T cells in the lungs of ARDS mice at 7 days after mMSCs transplantation. **a**–**d** The differentiation of Th17 and Treg in the lungs of LPS-induced ARDS mice was detected by flow cytometry (*n* = 3, *p < 0.05 compared with the control group; ^#^*p* < 0.05 compared with the ARDS group; ^δ^*p* < 0.05 compared with the LPS + mBM-MSC-NC group). **e** Representative flow cytometry analysis was shown for each treatment group. ARDS, acute respiratory distress syndrome; mMSCs, mouse mesenchymal stem cells; NC, normal control

The levels of IL-17A and IL-10 were measured in lung homogenates at 3 and 7 days after mMSCs transplantation by western blot. Compared with that in the ARDS group, IL-17A content was significantly decreased in the LPS + mBM-MSC and LPS + mBM-MSC-NC groups (*p* < 0.05). mMSCs overexpressing TGFβ1 further reduced the concentration of IL-17A in the lungs compared with that in the LPS + mBM-MSC-NC group (*p* < 0.05, Fig. 6a). Meanwhile, compared with that in the ARDS group, IL-10 content was significantly elevated in the LPS + mBM-MSC and LPS + mBM-MSC-NC groups (*p* < 0.05). mMSCs overexpressing TGFβ1 could further increase the concentration of IL-10 in the lungs compared with that in the LPS + mBM-MSC-NC group (*p* < 0.05, Fig. 6b). It was suggested that mMSCs overexpressing TGFβ1 could inhibit the expression of IL-17A while increasing IL-10 levels in the lungs of ARDS mice.

RETRACTED

**Fig. 6:** The effect of mMSCs overexpressing TGFβ1 on inflammatory factors in the lungs of ARDS mice. **a** The expression of the IL-17A and **b** IL-10 proteins in the lungs of all the experimental groups at 3 and 7 days after mMSCs administration was evaluated by western blot analysis (*n* = 3, *p < 0.05 compared with the control group; ^#^*p* < 0.05 compared with the ARDS group; ^δ^*p* < 0.05 compared with the LPS + mBM-MSC-NC group). ARDS, acute respiratory distress syndrome; mMSCs, mouse mesenchymal stem cells; NC, normal control

To further evaluate the inflammation in the lungs of ARDS mice, proinflammatory cytokines TNF-α, IL-1β, and IL-6 concentration in BALF of ARDS mice were also measured using ELISA. The expression of TNF-α, IL-1β and IL-6 in BALF were all significantly elevated in response to the LPS challenge (*p* < 0.0001). The treatment with mBM-MSC-TGFβ1 statistically decreased TNF-α, IL-1β, and IL-6 levels than the mBM-MSC-NC did at both 3 and 7 days (*p* < 0.05, Supplementary Figure 2A-C).

### Overexpression of TGFβ1 in mesenchymal stem cells improved the lung permeability of ARDS mice

The LWW/BW was calculated to evaluate lung oedema. The LWW/BW was significantly reduced in the LPS + mBM-MSC, LPS + mBM-MSC-NC, and LPS + mBM-MSC-TGFβ1 groups compared with that in the ARDS group at 3 and 7 days (*p* < 0.05, Fig. 7a).

**Fig. 7:** The effect of mMSCs overexpressing TGFβ1 on the permeability of LPS-induced lungs in mice. **a** Lung oedema was analysed by LWW/BW (*n* = 3, *p < 0.05 compared with the control group; ^#^*p* < 0.05 compared with the ARDS group). **b** Total protein and **c** albumin concentrations in bronchoalveolar lavage fluid were analysed by a mouse-specific ELISA kit to evaluate the permeability of the lung (*n* = 3, *p < 0.05 compared with the control group; ^#^*p* < 0.05 compared with the ARDS group; ^δ^*p* < 0.05 compared with the LPS + mBM-MSC-NC group). **d** Expression of the occludin protein in the lungs of all the experimental groups at 3 and 7 days after mMSCs administration was evaluated by western blot analysis (*n* = 3, *p < 0.05 compared with the control group; ^#^*p* < 0.05 compared with the ARDS group; ^δ^*p* < 0.05 compared with the LPS + mBM-MSC-NC group). ALB, albumin; ARDS, acute respiratory distress syndrome; ELISA, enzyme-linked immunosorbent assay; LWW/BW, lung wet weight/body weight; mMSCs, mouse mesenchymal stem cells; NC, normal control; TP, total protein

To evaluate whether mMSCs overexpressing TGFβ1 could alter the permeability of the lung, total protein and albumin concentrations in the BALF were measured by mouse-specific ELISAs. The total protein and albumin concentrations were significantly reduced in the LPS + mBM-MSC and LPS + mBM-MSC-NC groups compared with those in the ARDS group at both 3 and 7 days (*p* < 0.05). Significant decreases in the total protein and albumin concentrations were also observed in the LPS + mBM-MSC-TGFβ1 group compared with those in the LPS + mBM-MSC-NC group at 3 and 7 days (*p* < 0.05, Fig. 7b, c).

RETRACTED

Additionally, the occludin protein expression level increased significantly in the LPS + mBM-MSC and LPS + mBM-MSC-NC groups compared with that in the ARDS group (*p* < 0.05). A significant increase was also observed in the LPS + mBM-MSC-TGFβ1 groups compared to that in the ARDS group (*p* < 0.05), and the increase was much greater than that in the LPS + mBM-MSC-NC group (*p* < 0.05, Fig. 7d).

### Mesenchymal stem cells overexpressing TGFβ1 improved the pulmonary histopathology of lipopolysaccharide-induced ARDS mice

After LPS-induced lung injury, alveolar wall thickening, alveolar and interstitial inflammatory cell infiltration, haemorrhage, alveolar exudate, and oedema were observed in the lung tissues of ARDS group mice (Fig. 8a), and the Smith score for quantifying lung injury was also increased significantly (*p* < 0.05, Fig. 8b) in the ARDS group. However, compared to those in the ARDS group, histopathologic characteristics and the Smith score were alleviated at 3 and 7 days in the LPS + mBM-MSC and LPS + mBM-MSC-NC groups (*p* < 0.05, Fig. 8a, b). The effects were greater in the LPS + mBM-MSC-TGFβ1 group than in the LPS + mBM-MSC-NC group (*p* < 0.05, Fig. 8a, b).

**Fig. 8:** The effect of mMSCs overexpressing TGFβ1 on the histopathology of LPS-induced lung injury in mice. **a** Typical histopathological images of the lung tissues from mice of all the experimental groups at 3 and 7 days after LPS exposure (HE staining, × 50). **b** Lung injury score (Smith score) of the lung tissues from mice of all the experimental groups at 3 and 7 days after LPS challenge (*n* = 3 at each time-point for each group; *p < 0.05 compared with the control group; #*p* < 0.05 compared with the ARDS group; δ*p* < 0.05 compared with the LPS + mBM-MSC-NC group). ARDS, acute respiratory distress syndrome; mMSCs, mouse mesenchymal stem cells; NC, normal control

RETRACTED

### Effects of mMSCs overexpressing TGFβ1 on lung fibrosis in ARDS mice

To assess lung fibrosis, collagen deposition (which was stained blue) in lung tissue at 7 days after LPS challenge was analysed by Masson’s trichrome staining and was markedly increased in the ARDS group compared with that in the control group (*p* < 0.0001). The lung fibrosis score decreased significantly in the LPS + mBM-MSC, LPS + mBM-MSC-NC, and LPS + mBM-MSC-TGFβ1 groups compared to that in the ARDS group (*p* < 0.0001). Reduced collagen I and α-SMA mRNA was also observed after intervention with mBM-MSC, mBM-MSC-NC, or mBM-MSC-TGFβ1 compared with that in the ARDS group (*p* < 0.0001), but increased α-SMA mRNA was found in the LPS + mBM-MSC-TGFβ1 group compared with that in the LPS + mBM-MSC-NC group (*p* < 0.0001, Fig. 9a–d).

**Fig. 9:** The effect of mMSCs overexpressing TGFβ1 on lung fibrosis in ARDS mice. **a** Lung fibrosis was evaluated by Masson’s trichrome staining at 7 days after LPS exposure (× 200). A blue signal indicated positive staining for collagen, and a red signal represented muscle fibrosis and cellulose. **b** The quantification of lung fibrosis is shown as an Ashcroft score (*n* = 10, *p < 0.05 compared with the control group; ^#^*p* < 0.05 compared with the ARDS group). **c** Collagen I and **d** α-SMA mRNA in lungs was quantified by qRT-PCR (*n* = 3 at each time-point for each group; *p < 0.05 compared with the control group; ^#^*p* < 0.05 compared with the ARDS group; ^δ^*p* < 0.05 compared with the LPS + mBM-MSC-NC group). ARDS, acute respiratory distress syndrome; α-SMA, alpha smooth muscle actin; mMSCs, mouse mesenchymal stem cells; NC, normal control

### Effects of mMSCs overexpressing TGFβ1 on the survival of ARDS mice

Mice that received LPS challenge had a significantly decreased survival rate at 7 days compared with that of the control mice (*p* < 0.05). Although there was no significant difference in the survival rate in the LPS + mBM-MSC, LPS + mBM-MSC-NC, and LPS + mBM-MSC-TGFβ1 groups compared to that in the ARDS group, an upward trend was still found after mMSCs treatment (*p* > 0.05, Fig. 10).

RETRACTED

**Fig. 10:** Kaplan-Meier survival curves. Mice that received LPS challenge in each group were followed for 7 days after mMSCs administration (*n* = 18 for each group, *p < 0.05 compared with the control group)

## Discussion

Immunotherapy, one of the important treatments for ARDS, has not made any breakthroughs in the past two decades [18]. A large number of studies have shown that MSCs, multifunctional stem cells with low immunogenicity, could significantly improve the immunity state of ARDS in animal models [19, 20]. The mechanism is due mainly to the paracrine regulation of cell function and state by a variety of cytokines. TGFβ1, as a main paracrine cytokine of MSCs, could regulate the systemic immunity state by modulating the differentiation of T cells in ARDS. In our study, we first constructed mMSCs overexpressing TGFβ1, and the main findings were as follows. (1) Overexpressing TGFβ1 inhibited the proliferation of mMSCs during days 5–7 but had no effect on their differentiation or migration. (2) mMSCs overexpressing TGFβ1 decreased lung permeability and inflammatory cytokine levels and improved the histopathology of lung tissue and in ARDS mice. (3) mMSCs overexpressing TGFβ1 could significantly modulate the differentiation of T cells into Th17 and Treg while inhibiting the ratio of Th17 and Treg. IL-17A content was also decreased while IL-10 content was increased in the lungs of ARDS mice after treatment with mMSCs overexpressing TGFβ1. (4) mMSCs overexpressing TGFβ1 did not aggravate lung fibrosis in ARDS mice.

As an important part of adaptive immunity, T cell immunity is involved in the development of ARDS [21, 22]. Several studies have shown that specific regulation of T cell differentiation could improve the immunity and inflammation state of ARDS in animal models, resulting in prognosis improvement [21, 23, 24]. It was also found in our study that the regulation of T cell differentiation in patients with community-acquired pneumonia was directly related to their prognosis [25]. Th17 and Treg, as paired CD4^+^ T cell subsets, directly contribute to the prognosis of patients with ARDS [9]. At present, the regulation of Th17 and Treg differentiation depends mainly on antigen-presenting cells, cytokines, and intracellular signalling pathways [12]. However, TGFβ1, an important factor regulating T cell differentiation, had very low expression in MSCs. In our study, overexpression of TGFβ1 in mMSCs by lentivirus transduction significantly increased TGFβ1 mRNA and protein levels in the cells, as well as in the supernatant of culture media. However, there was no significant effect on the differentiation and migration of MSCs after transduction. The inhibited migration of mMSCs overexpressing TGFβ1 may be related to the involvement of TGFβ1 in the differentiation of MSCs via cell cycle regulation, which still needs further study.

RETRACTED

In this study, the therapeutic effect of MSCs after TGFβ1 transduction was significantly improved, due mainly to the better regulation of T cell differentiation in ARDS mice on day 3 and day 7 and reduced Th17/Treg ratio, thus balancing inflammatory cytokines in vivo. In our previous studies, specific regulation of inflammatory cytokines such as angiotensin-converting enzyme 2 (ACE2) or prostaglandin E2 (PGE2) in MSCs could also improve their therapeutic effects in ARDS animals, which paralleled the results of this study [10, 26]. In addition, a recent study also indicated that MSCs could prevent the differentiation of naive CD4^+^ T cells into Th17, inhibit the production of inflammatory cytokines by Th17, and induce the Treg phenotype in vitro [27]. However, in our study, the effect of MSCs overexpressing TGFβ1 on CD4^+^ T cells was mainly to increase the amount of Treg without reducing the number of Th17, which may be related to the animal status and detection methods. How to regulate Th17 and Treg differentiation specifically still needs further study in vitro.

TGFβ1 is also an important index of fibrosis and inflammation [28]. Despite this, pulmonary fibrosis in ARDS mice was also detected after MSCs transplantation [29]. According to Masson’s staining or specific mRNA expression, MSCs overexpressing TGFβ1 did not significantly increase pulmonary fibrosis in ARDS mice. In addition, our previous study also found that mMSCs could further improve the epithelial injury and pulmonary fibrosis of ARDS mice by increasing differentiation into type II epithelial cells through p130/E2F4 pathway [15], indicating that there might be no side effects related to MSCs transplantation.

This study still has several limitations. First, we induced ARDS by LPS treatment in mice. The murine model of ARDS induced by intratracheal LPS injection focuses only on inflammation in the lungs and cannot fully reflect the complexity of systematic inflammation seen in ARDS patients. Second, MSCs were only administered once intratracheally, and the mice were then sacrificed 3 and 7 days later, which may also not fully reflect the clinical application of such therapeutics; further studies focusing on different routes and doses for MSCs treatment are still needed.

## Conclusion

MSCs overexpressing TGFβ1 could regulate lung inflammation and attenuate lung injuries by modulating the imbalance of Th17/Treg in the lungs of ARDS mice.

RETRACTED

## Supplementary information

**Additional file 1: Supplementary Figure 1.** Flow cytometry identification of mMSCs overexpressing TGFβ1. Cell surface markers of mMSCs, including CD29, CD44, and CD105 were positive. Additionally, CD34 and CD45 of hematopoietic stem cells were negative. Red lines represent the isotype controls. FSC-A, forward scatter height; mMSCs, mouse mesenchymal stem cells; SSC-A, side scatter height.

**Additional file 2: Supplementary Figure 2.** Pro-inflammatory cytokines concentrations in bronchoalveolar lavage fluid of ARDS mice. A. TNF-α, B. IL-1β and C. IL-6 were analyzed by mouse specific ELISA to evaluate inflammation in lungs of ARDS mice. (*n* = 3, *p < 0.0001 compared with the Control group; #*p* < 0.05 compared with the ARDS group; δ*p* < 0.05 compared with the LPS + mBM-MSC-NC group).

**Additional file 3.**

## Data Availability

All data generated or analysed during this study are included in this published article.

## Abbreviations

ACE2: Angiotensin-converting enzyme 2
ALB: Albumin
ARDS: Acute respiratory distress syndrome
BALF: Bronchoalveolar lavage fluid
BSD: Blasticidin
CCK-8: Cell counting kit-8
CDS: Coding sequence
DMEM/F12: Dulbecco’s modified Eagle’s media/nutrient mixture F-12
EDTA: Trypsin-ethylenediaminetetraacetic acid
eGFP: Enhanced green fluorescent protein
ELISA: Enzyme-linked immunosorbent assay
FBS: Foetal bovine serum
FCM: Flow cytometry
IL: Interleukin
LPS: Lipopolysaccharide
LWW/BW: Lung wet weight/body weight
mBM-MSCs: Mouse bone marrow-derived mesenchymal stem cells
mBM-MSC-NC: Mouse bone marrow-derived mesenchymal stem cells carrying green fluorescent protein (normal control)
mBM-MSC-TGFβ1: Mouse bone marrow-derived mesenchymal stem cells carrying TGFβ1
mMSCs: Mouse mesenchymal stem cells
MOI: Multiplicity of infection
NS: Normal saline
PBS: Phosphate-buffered saline
PGE2: Prostaglandin E2
PVDF: Polyvinylidene difluoride
RIPA: Radioimmunoprecipitation assay buffer
ROIs: Regions of interest
SD: Standard deviation
SDS-PAGE: Sodium dodecyl sulfate-polyacrylamide gel electrophoresis
TBS: Tris-buffered saline
TBST: Tris-buffered saline with Tween-20
TGFβ1: Transforming growth factor β1
Th17: T helper 17 cells
TP: Total protein
TNF-α: Tumour necrosis factor-α
Treg: Regulatory T cells
WT: Wild-type
